# A network meta-analysis protocol of adjuvant chemotherapy for unresectable patients with advanced gastric cancer

**DOI:** 10.1097/MD.0000000000016108

**Published:** 2019-07-12

**Authors:** Long Li, Ling-yun Guo, Jie Mao

**Affiliations:** Department of First General Surgery, Lanzhou University Second Hospital, Lanzhou, China.

**Keywords:** 5-year survival rates, adjuvant chemotherapy, advanced gastric cancer, Bayesian, gastric cancer, perioperative mortalities, protocol, survival time, total mortalities

## Abstract

**Background:**

The treatment methods about surgery, chemotherapy, and radiation therapy were recommended for gastric cancer (GC) patients by National Comprehensive Cancer Network (NCCN) guidelines. However, for the advanced gastric cancer patients or with metastatic lesions who have lost their chance of surgery, the current adjuvant chemotherapy treatments are still controversial. Therefore, this network meta-analysis is mainly to assess the relative efficacy of different adjuvant chemotherapy regimens for advanced gastric cancer (AGC).

**Methods:**

In order to compare the relative efficacy among different adjuvant chemotherapy regimens for AGC patients, randomized controlled trials (RCTs) and non-RCTs were systematic searched in PubMed, Web of Science, Clinical Trials, Cochrane Library and Embase database. R-3.4.1 software will be used for data analysis. The risk of bias in RCTs and non-RCTs will be evaluated through the risk of bias tool from the Cochrane Handbook version 5.1.0 and non-randomized studies of interventions (ROBINS-I), respectively.

**Results and conclusion:**

The results of this network meta-analysis will evaluate the relative effectiveness and rank the interventions among all chemotherapy methods for unresectable AGC patients, and provide more evidence-based guidance in clinical practice.

**Protocol registration number:**

CRD42018111835.

## 1 Introduction

The latest Global cancer statistics 2018 showed that gastric cancer has become the fifth most prevalent cancer and the third leading cause of cancer-related death worldwide.^[1]^ The main reasons for the decline in the incidence and mortality of GC may be attributed to the popularity of gastroscopy and the diversity of treatment methods.^[2,3]^ However, the incidence of GC has been kept in a high level in China, and its 5-year survival rate is only 35.9%, far lower than South Korea's 68.9% and Japan's 60.3%.^[4]^ Due to the lack of effective screening, the majority of patients are in advanced stage at the initial diagnosis, and their 5-year survival rate is less than 30%, and the prognosis of unresectable AGC patients are more serious.^[5]^

According to the GC NCCN guidelines, radical gastrectomy is the standard treatment method and the chemotherapy, radiotherapy and biological immunotherapy are important adjuvant therapy methods.^[6]^ However, the first-line chemotherapy regimens recommended by the NCCN guidelines for unresectable AGC patients are various without clear indications, and the comparation of relative efficacy.^[5,7]^

Paired meta-analysis has the disadvantage of not being able to integrate all the information of chemotherapy methods from different original studies at the same time. Therefore, it is impossible to compare the pros and cons of different chemotherapy regimens. However, even if there was lacking of head-to-head comparisons, the network meta-analysis can also evaluate the relative effectiveness and rank the interventions among all chemotherapy methods for AGC patients, and provide more evidence-based guidance for clinical practice.^[8]^

The aim of this study is to evaluate the relative efficacy of different adjuvant treatments for AGC patients in the improvement of 1-, 2-, 3-year survival rates, survival time, short-term curative effects and the performance status (PFS) through this network meta-analysis.

## 2 Methods

### 2.1 Registration

This network meta-analysis protocol according to the preferred reporting items for systematic review and meta-analysis protocols (PRISMA-P) extension statement.^[9]^ Our protocol has been registered on the international prospective register of systematic review (PROSPERO) network. The registration number was CRD42018111835.

### 2.2 Ethics and dissemination

#### 2.2.1 Ethics issues

This network meta-analysis is a secondary research which based on some previously published data. Therefore, the ethical approval or informed consent was not required in this meta-analysis.

#### 2.2.2 Publication plan

This network meta-analysis will be published in a peer-reviewed journal.

### 2.3 Inclusion criteria

#### 2.3.1 Types of studies

RCTs and non-RCTs will be incorporated in this study without published year, publication status limitations.

#### 2.3.2 Types of participants

AGC Patients without age, gender, racial and region limitations, which were diagnosed and classified according to the NCCN guideline^[6]^;

#### 2.3.3 Types of interventions

According to different chemotherapy regimens, there are 7 interventions: only fluoropyrimidine, only paclitaxel/docetaxel, fluoropyrimidine (include fluorouracil or capecitabine) with oxaliplatin/cisplatin, paclitaxel/docetaxel with cisplatin/carboplatin, fluorouracil with irinotecan, modified DCF regimen (docetaxel, cisplatin/carboplatin/oxaliplatin, and fluorouracil), ECF or modified ECF regimen (epirubicin, cisplatin/oxaliplatin, and fluorouracil/capecitabine). Based on the different drugs in each intervention group, a more detailed subgroup analysis will be conducted to present the efficacy of different drugs.

#### 2.3.4 Type of outcomes

The primary outcomes are 1-, 2-, 3-year survival rates and overall survival. The secondary outcomes are short term efficacy according to Response Evaluation Criteria in Solid Tumors 1.1 (RECIST Criteria 1.1).

### 2.4 Information source

Five databases were searched as followings: PubMed, the Cochrane Library, Web of Science, Clinical Trials and EMBASE. The references of included articles and other relevant studies will be also tracked for additional supplement.

The retrieval keywords as followings: advanced gastric neoplasm, advanced gastric cancer, advanced stomach neoplasm, advanced stomach cancer, and adjuvant chemotherapy.

### 2.5 Data collection and analysis

#### 2.5.1 Data management

Endnote X7 software will be used for literature managing and records searching. A pilot-test will be conducted to ensure the inter-rater is reliability between the reviewers before the literature selection.

#### 2.5.2 Selection process

Two independent researchers will conduct a systematic search on above 5 databases according to the predetermined search strategy. In the case of the above-mentioned screening of documents and the extraction of data, if there is a disagreement, it will be resolved through discussion or assistance to a third reviewer. All the study selection process will be revealed in a flow diagram in accordance with the PRISMA guidelines.^[10]^

#### 2.5.3 Data collection process

Two independent researchers extracted data in the same predetermined table through the excel software. Any disagreements will be resolved by a third reviewer. The extraction data items as following: the first author, country, published year, the trial design, sample size, age, gender, regimen of adjuvant treatments, tumor pathological classification, TNM stage, 1-, 2-, 3-year survival rates, short-term effect (CR, PR, SD, PD), the PFS of patients, and some other outcomes of interest.

### 2.6 Quality of evidence assessment

According to Grading of Recommendations Assessment Development and Evaluation (GRADE), the quality of included studies will be assessed by the online guideline development tool (GDT, http://gdt.guidelinedevelopment.org/), and divided into 4 levels: high quality, moderate quality, low quality, and very low quality.^[11]^

### 2.7 Risk of bias individual studies

The risk of bias individual RCT studies will be evaluated from 7 specific domains (sequence generation, allocation concealment, blinding of participants and personnel, incomplete outcome data, selective reporting, and other bias and risk) on the basis of the Cochrane Handbook version 5.1.0.^[12]^ The methodological quality will be also evaluated as low risk, high risk, or unclear risk of bias in accordance with the criteria of the risk of bias judgment.^[13]^ According to the tool for assessing risk of bias in non-randomized studies of interventions (ROBINS-I),^[14]^ the risk of bias of non-randomized studies which included in this network meta-analysis will be estimated as following: confounding, the selection of participants, intervention classification, bias due to deviations from intended interventions, missing data, the measurement of outcomes, the selection of the result reporting, and overall risk bias. The risk of bias will be divided into five parts as following: low, moderate, serious, critical risk of bias, and no information. All the assessment of risk of bias will be performed and finished by 2 researchers independently, any disagreements will be resolved through a third researcher.

### 2.8 Geometry of the network

The function of *‘forest.netmeta’* of R-3.4.1 (R Foundation for Statistical Computing, Vienna, Austria) will be used to draw network plots to describe and present the geometry of different chemotherapy regimens. The nodes and edges will be used to reveal the head-to-head comparisons among interventions.

### 2.9 Pairwise meta-analysis

The extracted data of all the included studies will be summarized and presented through Excel 2010. Pairwise meta-analysis will be conducted R-3.4.1 software. The statistical heterogeneity among included studies will be assessed by Higgins *I*^*2*^ statistic (large, if *I*^*2*^> 50%; medium if 25% < *I*^*2*^ ≥ 50%; and small if 0 ≤ *I*^*2*^ ≥ 25%).^[15]^ Fixed-effect model analysis will be performed, if there is no evidence showed heterogeneity; Otherwise, random-effect model analysis will be chosen after excluding the sources of heterogeneity.

### 2.10 Network meta-analysis

The ‘*netmeta*’ version 0.9–8 of R-3.4.1 software will be used to perform a network meta-analysis to synthesize direct and indirect evidence for assessing the therapeutic effect among different adjuvant chemotherapy regimens for AGC patients who have lost the surgery opportunities.^[16]^ Inconsistency between direct and indirect comparisons will be assessed by the node splitting method when a loop connecting three arms existed. The treatment effects of different chemotherapy regimens for AGC patients will be ranked by the *P* scores which based on the point estimates and standard errors of the network assessment.

### 2.11 Other analyses

#### 2.11.1 Subgroup and sensitivity analyses

Subgroup analyses, which are designed for age, gender, region and different adjuvant chemotherapy regimens, will be used to find the possible sources on account of a possibility of significant heterogeneity or inconsistency.

#### 2.11.2 Publication bias

Egger graph and Begg graph will be drawn by the STATA V.12.0 software to identify whether this meta-analysis will have a publication bias.

## Author contributions

LL, GLY planed and designed the research; MJ and LL tested the feasibility of the study; MJ and LL wrote the manuscript; all authors approved the final version of the manuscript.

**Conceptualization:** Jie Mao, Lingyun Guo.

**Data curation:** Long Li.

**Investigation:** Long Li.

**Methodology:** Lingyun Guo.

**Project administration:** Jie Mao, Lingyun Guo.

**Resources:** Jie Mao, Lingyun Guo.

**Software:** Long Li.

**Supervision:** Lingyun Guo.

**Validation:** Jie Mao.

**Writing – original draft:** Long Li.

**Writing – review & editing:** Jie Mao.

## References

[1] BrayFFerlayJSoerjomataramI Global cancer statistics 2018: GLOBOCAN estimates of incidence and mortality worldwide for 36 cancers in 185 countries. CA Cancer J Clin 2018.10.3322/caac.2149230207593

[2] LHkMDHH Randomized trial of adjuvant chemotherapy with mitomycin, Fluorouracil, and Cytosine arabinoside followed by oral Fluorouracil in serosa-negative gastric cancer: Japan Clinical Oncology Group 9206-1. J Clin Oncol 2003;21:2282–7.1280532710.1200/JCO.2003.06.103

[3] SarelaAILefkowitzRBrennanMF Selection of patients with gastric adenocarcinoma for laparoscopic staging. Am J Surg 2006;191:134–8.1639912410.1016/j.amjsurg.2005.10.015

[4] BouzbidSHamdi-ChérifMZaidiZ Global surveillance of trends in cancer survival 2000-14 (CONCORD-3): analysis of individual records for 37 513 025 patients diagnosed with one of 18 cancers from 322 population-based registries in 71 countries. Lancet 2018.10.1016/S0140-6736(17)33326-3PMC587949629395269

[5] De-VitaFGiulianiFGaliziaG Neo-adjuvant and adjuvant chemotherapy of gastric cancer. Ann Oncol 2007;18:120–3.10.1093/annonc/mdm23917591804

[6] AjaniJABentremDJBeshS Gastric cancer, version 2.2013: featured updates to the NCCN Guidelines. J Natl Compr Canc Netw 2013;11:531–46.2366720410.6004/jnccn.2013.0070

[7] AjaniJAD’AmicoTABaggstromM Gastric Cancer, Version 5.2017, NCCN clinical practice guidelines in oncology. J Natl Compr Canc Netw 2017;14:1286.

[8] BafetaATrinquartLSerorR Reporting of results from network meta-analyses: methodological systematic review. BMJ 2014;348(mar11 5):g1741.2461805310.1136/bmj.g1741PMC3949412

[9] ShamseerLMoherDClarkeM Preferred reporting items for systematic review and meta-analysis protocols (PRISMA-P) 2015: elaboration & explanation. BMJ 2015;349:g7647–17647.10.1136/bmj.g764725555855

[10] MoherDLiberatiATetzlaffJ Preferred reporting items for systematic reviews and meta-analyses: The PRISMA statement. Int J Surg 2010;8:336–41.2017130310.1016/j.ijsu.2010.02.007

[11] PuhanMASchünemannHJMuradMH A GRADE Working Group approach for rating the quality of treatment effect estimates from network meta-analysis. BMJ 2014;349(sep24 5):g5630.2525273310.1136/bmj.g5630

[12] HigginsJPTGreenS Cochrance Handbook for Systematic Reviews of Interventions Version 5.1.0 [EB/OL]. The Cochrane Collaboration. 2011 http://www.cochrane-handbook.org [Accessed on May 16, 013]

[13] HigginsJPT ADSterneJAC Chapter 8: Assessing risk of bias in included studies. Cochrane Handbook for Systematic Reviews of Interventions Version 5.1.0 (updated March 2011). The Cochrane Collaboration. 2011.

[14] SterneJAHernánMAReevesBC ROBINS-I: a tool for assessing risk of bias in non-randomised studies of interventions. BMJ 2016;355:i4919.2773335410.1136/bmj.i4919PMC5062054

[15] HigginsJPThompsonSG Quantifying heterogeneity in a meta-analysis. Stat Med 2002;21:1539–58.1211191910.1002/sim.1186

[16] John Wiley & Sons, Ltd, GurusamyKS Management strategies for pancreatic pseudocysts: a network meta-analysis. 2014.

